The article "Construction and Analysis of Discrete System Dynamic Modeling of Physical Education Teaching Mode Based on Decision Tree Algorithm" was published in 2022. Journal: Comput Intell Neurosci.

# Construction and Analysis of Discrete System Dynamic Modeling of Physical Education Teaching Mode Based on Decision Tree Algorithm

**DOI:** 10.1155/2022/2745146

**Published:** 2022-07-19

**Authors:** Caixia Wang, Xiaoyun Wei, Aiqian Yang, Haiyan Zhang

**Affiliations:** ^1^College of Physical Education, Handan University, Hebei 056000, China; ^2^College of Physical Education, Hengshui University, Hebei 056000, China

## Abstract

Physical education is not only an important part of national education but also one of the important means to improve the physical quality of students and citizens. Therefore, the reform of physical education is of great significance to the development of physical education. With the application of data mining technology in the field of physical education, the scale of relevant data increases rapidly. The traditional data analysis methods cannot meet the needs of physical education data analysis. Traditional data analysis methods still have many basic problems to be solved. For example, the professionalism of the structural model and standardization of formal expression are dwarfed by the forefront of the world. There are few real valuable data in the database, and the referentiality is not guaranteed. Therefore, this study puts forward the construction and analysis of discrete system dynamic modeling of physical education teaching mode based on the decision tree algorithm. Through the decision tree algorithm, this study analyzes the data related to physical education and constructs the physical education decision tree system according to the analysis structure. The test results show that the primary influencing factor of physical education teaching is the number of students participating in sports competitions, and the secondary influencing factors are students' liking and teachers' skill level. In addition, teachers' adjustment of physical education teaching contents and methods according to the analysis results of decision tree is conducive to improving students' physical education performance.

## 1. Introduction

With the rapid development of computer technology, computer technology has been applied to various fields. With the development of various network technologies, the development of computer technology has also brought broad prospects to the modernization of physical education. It also brings unprecedented challenges and opportunities to educators. When the network changes people's way of work, study, thinking, and communication at an amazing speed, the traditional classroom, textbook, and teacher centered teaching mode has also been impacted by the computer network, and the physical education mode should be reformed with the changes of the times. If the traditional teaching mode and scientific teaching method cannot be updated in time, it will cause some outdated teaching methods cannot be updated in the field of physical education. As an important part of the education system, physical education not only has commonness with other educational disciplines but also has its own characteristics. Sports itself is the integration of humanities and natural sciences. These determine that the physical education discipline is an open, developing, and innovative system.

The article "Construction and Analysis of Discrete System Dynamic Modeling of Physical Education Teaching Mode Based on Decision Tree Algorithm" was published in 2022. Journal: Comput Intell Neurosci.

Physical education is an important part of national quality education. It can not only help students effectively enhance their physique and improve their physical quality but also help students adjust their emotions and improve their psychological state, so as to maintain their physical and mental health [1]. At the same time, the practical course in physical education teaching is an effective and rapid method for students to understand and master corresponding knowledge and skills. With the continuous improvement of computer technology and the implementation of the domestic education reform system, great changes have taken place in the teaching content and teaching mode of physical education, and the evaluation standard of physical education teaching quality has also changed [2]. Therefore, it has become a research hotspot of physical education reform to understand the influencing factors of physical education teaching quality through physical education teaching evaluation and improve targeted and effective physical education teaching. Modern teaching equipment and management system have produced a large number of relevant data in the application of physical education. If the previous manual means are used to analyze and process these data, it will produce large time cost and labor cost [3]. In addition, it is difficult to quickly analyze the relationship between physical education teaching data in a short time by manual means and determine the factors affecting the quality of physical education teaching according to different courses. Data mining can process and analyze massive data according to the given target task, combined with the technology of machine learning, database, statistics, and other disciplines, and present the effective information that people can understand, extracted from massive data, so as to provide reference statistical analysis data results for people's decisions.

Therefore, this study puts forward the construction and analysis of discrete system dynamic modeling of physical education teaching mode based on the decision tree algorithm, in which the decision tree algorithm is an inductive learning algorithm that can reason in a group of irregular and sequential examples in data mining technology and summarize the expression form of decision tree. Through the construction of the decision tree algorithm to find the potential relationship between various factors of physical education teaching and teaching mode, the corresponding teaching side improvement strategies are obtained. This study is mainly divided into three parts. The first part expounds the development and current situation of data mining. The second part is the construction of the physical education teaching model based on the decision tree algorithm. The third part tests and analyzes the results of the physical education teaching model system based on the decision tree algorithm.

The article "Construction and Analysis of Discrete System Dynamic Modeling of Physical Education Teaching Mode Based on Decision Tree Algorithm" was published in 2022. Journal: Comput Intell Neurosci.

## 2. Related Work

The popularity of the Internet makes the data in databases in various fields grow at a geometric multiple rate, and the technology of data mining and analysis is also developing [4]. In the era of big data, data mining has been applied in the field of education, which provides data support for the improvement of education and has achieved good results. Some foreign scholars have conducted data mining and corresponding in-depth analysis and research on the education data in the ten years since 1995, concluded the necessity and importance of corresponding research on student data in the field of education, and provided research and analysis results for students, education-related workers, and managers [5]. In addition, foreign scholars apply data mining technology to the analysis of students' classroom behavior, correct students' wrong behavior in the classroom through the results of data analysis, and formulate targeted teaching measures to help students correct misconduct and improve their grades [6]. In the process of research, some scholars found that there is a certain relationship between students' academic performance and the nature of the school, and the level of socioeconomic status has different effects on the performance of boys and girls [7]. Through the regression analysis algorithm in data mining technology, some scholars have shown that students' parents and their family income are closely related to students' academic performance [8]. Wang used analysis of variance to conclude that students who participate in after-school activity groups usually have better grades. Other scholars have studied the relationship between students' performance and achievement through data mining technology and hope that this research result can provide some guidance for scaffolding teaching [9].

Compared with foreign countries, the application of data mining technology in the field of education in China was about 2001. It was not until the creation of the International Journal of Educational Data Mining in 2009 that China gradually paid attention to the application of data mining technology in the field of education [10]. By 2013, education data mining in its infancy has ushered in an important turning point, and then, China's education data mining began to enter the stage of rapid development. Therefore, compared with foreign countries, the development time of educational data mining in China is relatively short, and there is a certain gap in the breadth and depth of research. In recent years, the research on educational data mining in student modeling, achievement prediction, and learning resource recommendation system is gradually increasing. Based on the research on the current distance education system, some scholars proposed to make up for the deficiency of the distance education system framework through data mining technology, so that network education can give full play to its advantages and continuously improve the quality and level of network teaching [11]. Other scholars have deeply analyzed and elaborated the satisfaction data of college students obtained through data mining technology from the perspective of learning, mined the influencing characteristic factors of college students' learning characteristics and behavior on satisfaction, and verified and analyzed the relationship between them. Their research results provide effective data reference for talent training in colleges and universities [12]. Some scholars analyze the data information generated by students in the process of online English learning through the decision tree algorithm in the data mining algorithm to predict the test results of online English and provide corresponding suggestions and strategies for improving students' English test clearance rate [13]. In addition, some scholars use the ID3 decision tree algorithm to manage and analyze the results of business English practice examination and put forward targeted improvement evaluation and suggestions on the course content according to the data analysis results, thus promoting the reform of teaching quality evaluation management [14]. But at present, the research on data mining in physical education teaching is still relatively few, and it is still in the preliminary development stage, so more research and practice are needed.

The article "Construction and Analysis of Discrete System Dynamic Modeling of Physical Education Teaching Mode Based on Decision Tree Algorithm" was published in 2022. Journal: Comput Intell Neurosci.

## 3. Construction of the Physical Education Teaching Model Based on the Decision Tree Algorithm

### 3.1. Design of the Physical Education Teaching Mode System Based on the Decision Tree Algorithm

Physical education teaching includes not only theoretical knowledge teaching but also practical teaching, which affect and assist each other. Therefore, the application of data mining technology in the field of physical education can count and analyze a large number of relevant curriculum data and realize the analysis and query of students' physical education achievements. According to the results of students' performance analysis of different sports, we can reasonably plan the physical education curriculum, make the physical education teaching mode conform to students' actual physical quality and interests, and finally improve students' enthusiasm to participate in physical education curriculum and carry out personalized physical education on the basis of basic teaching. In physical education class, use light, lively, and interesting music or games to replace the preparation of boring and repeated running. It can create a relaxed and harmonious teaching atmosphere, improve students' learning enthusiasm, and receive good teaching results. Stimulate interest in classroom teaching; teachers should give full play to their language advantages and use enlightening questions, which will effectively arouse students' interest in exploring new causes and arouse students' desire for knowledge. As shown in Figure 1, it is the system framework of physical education teaching mode based on the decision tree algorithm.

In the process of physical education teaching, we need to carry out the fragment teaching of physical education theoretical knowledge points and then master and apply the knowledge points in combination with physical education practice. This requires teachers to explain the knowledge points of each part through horizontal, vertical, systematic, and expansionary ways in physical education teaching. Students choose one or a combination of multiple ways to learn according to their own actual situation and objective environment. In this way, teachers can also carry out personalized teaching according to the learning situation of different students and realize classified teaching. Decision analysis is an important part of the physical education teaching mode system based on the decision tree algorithm. The result of decision analysis is based on students' learning state, physical education teaching content and methods, and knowledge points. It is a long-term dynamic process of data statistics, analysis, and mining. Therefore, the data scale of decision analysis is the decisive factor affecting the accuracy and reliability of decision analysis results, and the decision results will change with the continuous accumulation of data and the change of environmental conditions.

The decisive factors affecting the accuracy and reliability of decision analysis results are the stability of the environment. When the environment is relatively stable, the decision-making made by the organization for similar embryos in the past has a high reference value because the environment faced in the past decision-making is similar to that at present. Market structure: decision-making usually focuses on how to pay close attention to the movements of competitors. The degree of informatization of the organization: organizational decision makers with a high degree of informatization usually have more advanced decision-making means.

The article "Construction and Analysis of Discrete System Dynamic Modeling of Physical Education Teaching Mode Based on Decision Tree Algorithm" was published in 2022. Journal: Comput Intell Neurosci.

Figure 2 shows the application structure of the decision base of physical education teaching mode based on the decision tree algorithm.

### 3.2. Thinking and Construction of Decision Tree Application

The most important algorithm in the decision tree generation algorithm is ID3 interactive diesel version 3, which was first proposed by Quinlan. Its basic idea is to use mutual information (or information gain) in information theory. As a measure of the classification and discrimination ability of decision attributes, the decision node attributes are selected. In the ID3 algorithm, the concept of entropy in information theory is applied to select the attributes of decision nodes, and the decision tree is established through the attributes with maximum information gain (or maximum entropy compression). The node attributes selected in this way ensure that the decision tree has the minimum number of branches and the minimum redundancy 2.

Decision tree is to recursively search the classification rules in irregular cases from top to bottom through information gain in the form of tree view. In the process of decision tree data classification, it is necessary to analyze and test the obtained dataset and construct the data classification model of physical education teaching mode according to the results. Each decision node of the decision tree is a test point for attribute value comparison. Each branch is a test output of different attribute values, and each leaf node represents the obtained conclusion. The branches formed by the decision tree reflect the data in the training set, that is, in addition to the normal classification, there are abnormal conditions, which is easy to cause excessive data. Therefore, the decision tree needs to be pruned accordingly to remove the abnormal branches, so as to ensure the accuracy of the results. The general idea of the application of decision tree in physical education teaching mode is to construct a decision tree containing the attribute values of each index according to the data of physical education teaching mode and obtain the important influencing factors of physical education teaching by sorting the given index set.

The article "Construction and Analysis of Discrete System Dynamic Modeling of Physical Education Teaching Mode Based on Decision Tree Algorithm" was published in 2022. Journal: Comput Intell Neurosci.

Decision tree strategy: divide and rule from top to bottom.

(i) The recursive process from root to leaf finds a “partition” attribute at each intermediate node
  - Start: build the root node. All training data are placed in the root node, and - optimal features are selected. According to this feature, the training dataset is divided into subsets and entered into subnodes.
  - All subsets are recursively divided according to the attributes of internal nodes
  - If these subsets can be classified basically correctly, build leaf nodes and distribute these subsets to corresponding leaf nodes
  - Each subset is divided into leaf nodes. In this way, a decision tree is generated.

Suppose that the two-dimensional structure data sample set *L* contains three knowledge point attribute fields and one teaching means attribute field, each knowledge point contains different attribute sets, that is, the knowledge point *K*_1_ is divided into three levels and expressed as {*A*_1_, *A*_2_, *A*_3_}, the knowledge point *K*_2_ is divided into two levels and expressed as {*B*_1_, *B*_2_}, the knowledge point *K*_3_ is divided into three levels and expressed as {*C*_1_, *C*_2_}, and the physical education teaching means include two ways and expressed as {*T*_1_, *T*_2_}. If the attribute field scale of the sample collection is *n* and an attribute field of the knowledge point is *K*_*i*_ and *i* ∈ {1,2,…, *n*}, the corresponding information entropy is shown in the following formula:

(1) $$\begin{array}{c} I\left(K_{i}\right)=-\sum_{i=1}^{n}p_{i}\log\;p_{i}, \end{array}$$

where*p*_*i*_ in the formula represents the probability of occurrence of corresponding attribute value, and each field is independent of each other.

Let |*T*_*i*_| represent the scale of *T*_*i*_; then, the information entropy of field *L* in sample set *T* is shown in the following formula:

(2) $$\begin{array}{c} I\left(T\right)=\left(-\frac{\left|T_{1}\right|}{\left|T\right|}\log_{2}\frac{\left|T_{1}\right|}{\left|T\right|}\right)+\left(-\frac{\left|T_{2}\right|}{\left|T\right|}\log_{2}\frac{\left|T_{2}\right|}{\left|T\right|}\right). \end{array}$$

Let |*T*_*i*_^*A*_*i*_^| represent the scale of the field corresponding to *A*_*i*_; then, the information gain of knowledge point *K*_1_ is shown in the following formula:

(3) $$\begin{array}{c} I\left(A_{i}\right)=\left(-\frac{\left|T_{1}^{A_{i}}\right|}{\left|T_{1}^{A_{i}}\right|+\left|T_{2}^{A_{i}}\right|}\log_{2}\frac{\left|T_{1}^{A_{i}}\right|}{\left|T_{1}^{A_{i}}\right|+\left|T_{2}^{A_{i}}\right|}\right)+\left(-\frac{\left|T_{2}^{A_{i}}\right|}{\left|T_{1}^{A_{i}}\right|+\left|T_{2}^{A_{i}}\right|}\log_{2}\frac{\left|T_{2}^{A_{i}}\right|}{\left|T_{1}^{A_{i}}\right|+\left|T_{2}^{A_{i}}\right|}\right). \end{array}$$

The income of knowledge point *K*_1_ is shown in the following formula:

(4) $$\begin{array}{c} E\left(K_{1}\right)=\frac{\left|A_{1}\right|}{\left|K_{1}\right|}I\left(A_{1}\right)+\frac{\left|A_{2}\right|}{\left|K_{2}\right|}I\left(A_{2}\right)+\frac{\left|A_{3}\right|}{\left|K_{3}\right|}I\left(A_{3}\right). \end{array}$$

The gain is shown in the following formula:

(5) $$\begin{array}{c} G\left(K_{1}\right)=I\left(T\right)-E\left(K_{1}\right). \end{array}$$

Similarly, if the *T*_1_ scale of the attribute value *B*_*i*_ in the knowledge point *K*_2_ is expressed as |*T*_1_^*B*_*i*_^| and the *T*_2_ scale is expressed as |*T*_2_^*B*_*i*_^|, the information gain is shown in the following formula:

(6) $$\begin{array}{c} I\left(B_{i}\right)=\left(-\frac{\left|T_{1}^{B_{i}}\right|}{\left|T_{1}^{B_{i}}\right|+\left|T_{2}^{B_{i}}\right|}\log_{2}\frac{\left|T_{1}^{B_{i}}\right|}{\left|T_{1}^{B_{i}}\right|+\left|T_{2}^{B_{i}}\right|}\right)-\left(-\frac{\left|T_{2}^{B_{i}}\right|}{\left|T_{1}^{B_{i}}\right|+\left|T_{2}^{B_{i}}\right|}\log_{2}\frac{\left|T_{2}^{B_{i}}\right|}{\left|T_{1}^{B_{i}}\right|+\left|T_{2}^{B_{i}}\right|}\right). \end{array}$$

The income of knowledge point *K*_2_ is shown in the following formula:

(7) $$\begin{array}{c} E\left(K_{2}\right)=\frac{\left|B_{1}\right|}{\left|K_{1}\right|}I\left(B_{1}\right)+\frac{\left|B_{2}\right|}{\left|K_{2}\right|}I\left(B_{2}\right). \end{array}$$

The gain is shown in the following formula:

(8) $$\begin{array}{c} G\left(K_{2}\right)=I\left(T\right)-E\left(K_{2}\right). \end{array}$$

Let the *T*_1_ scale of the attribute value *C*_*i*_ in the knowledge point *K*_3_ be expressed as |*T*_1_^*C*_*i*_^|, and the *T*_2_ scale be expressed as |*T*_2_^*C*_*i*_^|, and its information gain is shown in the following formula:

(9) $$\begin{array}{c} I\left(C_{i}\right)=\left(-\frac{\left|T_{1}^{C_{i}}\right|}{\left|T_{1}^{C_{i}}\right|+\left|T_{2}^{C_{i}}\right|}\log_{2}\frac{\left|T_{1}^{C_{i}}\right|}{\left|T_{1}^{C_{i}}\right|+\left|T_{2}^{C_{i}}\right|}\right)-\left(-\frac{\left|T_{2}^{C_{i}}\right|}{\left|T_{1}^{C_{i}}\right|+\left|T_{2}^{C_{i}}\right|}\log_{2}\frac{\left|T_{2}^{C_{i}}\right|}{\left|T_{1}^{C_{i}}\right|+\left|T_{2}^{C_{i}}\right|}\right). \end{array}$$

The income of knowledge points *K*_3_ is shown in the following formula:

(10) $$\begin{array}{c} E\left(K_{3}\right)=\frac{\left|C_{1}\right|}{\left|K_{3}\right|}I\left(C_{1}\right)+\frac{\left|C_{2}\right|}{\left|K_{3}\right|}I\left(C_{2}\right). \end{array}$$

The gain is shown in the following formula:

(11) $$\begin{array}{c} G\left(K_{3}\right)=I\left(T\right)-E\left(K_{3}\right). \end{array}$$

Then, calculate and compare the results according to the attribute values contained in the corresponding knowledge points. For example, the results are shown in the following formula:

(12) $$\begin{array}{c} G\left(K_{2}\right)>G\left(K_{1}\right)>G\left(K_{3}\right). \end{array}$$

It means that among the physical education teaching knowledge points in the sample set, the information gain of knowledge point *K*_2_ is the highest and the information gain of knowledge point *K*_3_ is the lowest. Therefore, the tree root of the physical education teaching decision tree is knowledge point *K*_2_, which is constructed on this basis. In Figure 3, the frame diagram of physical education teaching decision tree based on knowledge point *K*_2_ is shown.

The article "Construction and Analysis of Discrete System Dynamic Modeling of Physical Education Teaching Mode Based on Decision Tree Algorithm" was published in 2022. Journal: Comput Intell Neurosci.

According to the node path of the above decision tree, build a rule with the leaf node attribute value *T* as the rule tail and the nonleaf node attribute value *K*_1_∧*K*_2_∧*K*_3_ as the rule head and obtain the probability of *T* under the rule, that is, confidence *λ*. For example, the rule that the size of knowledge points is three is shown in the following formula:

(13) $$\begin{array}{c} K_{1}\wedge K_{2}\wedge K_{3}\Rightarrow T,\lambda . \end{array}$$

The corresponding confidence is shown in the following formula:

(14) $$\begin{array}{c} \lambda =\frac{P_{r}\left(k_{1}\cup k_{2}\cup k_{3}\cup T\right)}{P_{r}\left(k_{1}\cup k_{2}\cup k_{3}\right)}, \end{array}$$

where *P*_*r*_(*k*_1_ ∪ *k*_2_ ∪ *k*_3_ ∪ *T*) in the formula represents the probability value of the corresponding four attributes and *P*_*r*_(*k*_1_ ∪ *k*_2_ ∪ *k*_3_) represents the probability value of the corresponding three attributes.

The rule that can be obtained according to the physical education decision tree is not the only one, and the physical education teaching method can be selected according to the rule. For example, when the knowledge point 1 is *A*_1_, the knowledge point 2 is *B*_1_, and the physical education teaching method is *T*, the confidence *λ* expression is shown in the following formula:

(15) $$\begin{array}{c} K_{1}\left(A_{1}\right)\wedge K_{2}\left(B_{1}\right)\Rightarrow T\left(T_{1}\right),\lambda . \end{array}$$

## 4. System Test of Physical Education Teaching Mode Based on the Decision Tree Algorithm

In this study, 350 students in a certain university are randomly selected as the test objects of the physical education teaching mode system based on the decision tree algorithm. A variety of data collection methods are adopted to collect the basic information of students, and a physical education student database is constructed. Among them, the basic information of students has four basic indicators including students' grade, gender, intelligence level, and physical quality. At the same time, it also makes investigation and data statistics on students' physical education achievements, their love for physical education courses, current physical education teaching contents and methods, their participation in physical education competitions, and the evaluation of the physical education teaching effect. As shown in Figure 4, it is the statistics of eight attribute status of some groups of the training set of analysis variables selected by the test. Among them, the students' intelligence level, physical quality, and physical performance are divided into four levels, namely, unqualified, qualified, good, and excellent, which are expressed by the values of 0, 1, 2, and 3, respectively. Students' liking for physical education teaching is divided into like and dislike, that is, the numerical value 1 indicates like and 2 indicates dislike. The number of times students participate in sports competitions is divided into three levels, that is, they have not participated, participated once or twice, and participated more than three times, which are expressed by the values 1, 2, and 3, respectively. Physical education teaching means are also divided into three levels, that is, one teaching means, two to three teaching means, and more than three teaching means. The subtable is expressed in 1, 2, and 3. Teachers' skill levels are divided into national level, level I, and level II, which are expressed by the values 3, 2, and 1, respectively.

The article "Construction and Analysis of Discrete System Dynamic Modeling of Physical Education Teaching Mode Based on Decision Tree Algorithm" was published in 2022. Journal: Comput Intell Neurosci.

When the number of samples is small but the number of features is large, the decision tree is easy to over fit. For one thing, if the number of samples is more than the number of features, it will be easier to establish a robust model. When there are many features, PCA (principal component analysis), ICA (independent component analysis), and feature selection are preferred. Models that do not need data preprocessing are decision tree, random forest, and ICA. Because they do not care about the value of variables, they only care about the distribution of variables and the conditional probability between variables.

Remove the samples in the unqualified training set, set the remaining samples to the random seed mode, and select the sampling mode as random, in which 80% of the effective information is randomly selected as the training sample and the remaining 20% as the test sample. The training sample is applied to the construction of influencing factors of the physical education decision tree model. The test sample is to test and evaluate the physical education teaching mode system based on the decision tree algorithm. In this study, C5 decision tree software is selected to realize the node, and the attribute of branch node is the information gain rate with the highest and greater than or equal to the average value of all attributes. In Figure 5, the information gain and information gain rate of physical education decision tree are shown.

The article "Construction and Analysis of Discrete System Dynamic Modeling of Physical Education Teaching Mode Based on Decision Tree Algorithm" was published in 2022. Journal: Comput Intell Neurosci.

As shown in Figure 6, it is the decision tree of physical education teaching mode. It can be seen from the figure that the decision-making of physical education teaching mode takes the number of students participating in physical competitions as the root node, which shows that this factor is the most important factor affecting students' physical education performance. The number of students participating in sports competitions shows that students' sports achievements are in a good state and students' achievements are closely related to sports teaching mode. With the increase of the number of students participating in sports competitions, the excellent rate of sports achievements continues to increase, and the recognition of sports teaching mode will also increase. There are two main reasons for this. On the one hand, in the process of preparing for the competition, PE teachers will carry out targeted teaching and practice according to the characteristics of different students and help students improve the proficiency and accuracy of basic sports actions in repeated practice, which lays an important core foundation for students to participate in sports competitions. At the same time, in the process of participating in the competition, students can also have a new understanding of the basic sports skills and movements they have mastered from multiple angles, and the referees and PE teachers can guide students to observe the movements of high-level athletes, which is conducive to improving students' deeper understanding of the participating sports. It can effectively improve the completion ability and degree of students' sports technical movements. The replay after the competition is also a kind of feedback information for students' learning, which can help students understand their own shortcomings and point out the direction for subsequent exercises. At the same time, teachers can also find the shortcomings of physical education teaching content and teaching mode. Improve physical education teaching according to students' characteristics and current situation. Another reason is that sports competition is a physical education teaching method conducive to cultivating students' on-the-spot performance. Different from the daily physical education teaching environment, sports competition is relatively strange and complex for students, which is easy to affect students' psychological state. This kind of influence may be positive or negative, and the resulting emotions also have positive and negative effects. When participating in sports competitions, students need to actively adjust themselves, overcome the impact of environmental changes, and maintain their stable psychological state, so as to play a good on-the-spot performance ability in the competition.

The article "Construction and Analysis of Discrete System Dynamic Modeling of Physical Education Teaching Mode Based on Decision Tree Algorithm" was published in 2022. Journal: Comput Intell Neurosci.

The influential factor in the decision tree of physical education teaching mode is the students' liking for physical education teaching and the technical level of physical education teachers. Different PE teachers have different teaching styles and teaching methods. Students like the teaching of different PE teachers differently, and their ability to accept the teaching content is also different. Therefore, students' final PE scores are different. Generally, among the students taught by the same PE teacher, the students who like the PE teacher's teaching content and method have higher scores than the students who do not like and have low acceptance ability. Therefore, in the improvement of physical education teaching mode, we should pay attention to cultivating students' interest in physical education and increasing students' enthusiasm in learning physical education teaching content. There is also a close relationship between teachers' technical level and physical education teaching mode. Physical education teachers with higher technical level can better master the shortcomings of students' basic sports technology and action in the process of teaching, so as to give corresponding guidance and correction.

In addition to the above influencing factors, the diversity of PE teachers' teaching means, the number of PE teaching hours, and students' own physical quality will also affect the effect of PE teaching. The understanding level of different students can be divided into high and low. Teachers who use diversified teaching methods in physical education teaching can help students understand and learn the basic sports knowledge, actions, and skills from different angles, so as to improve students' physical education performance. In addition to learning theoretical knowledge, basic sports movements and skills also need repeated practice. Therefore, a reasonable physical education teaching time can provide students with the necessary opportunities for sports action technology practice, so as to improve students' performance. At the same time, students will also find their own problems in the process of practice and give timely feedback to physical education teachers, and teachers can find the places where their physical education teaching content needs to be strengthened according to students' feedback.

The article "Construction and Analysis of Discrete System Dynamic Modeling of Physical Education Teaching Mode Based on Decision Tree Algorithm" was published in 2022. Journal: Comput Intell Neurosci.

As shown in Figure 7, the results of students are compared after PE teachers adjust PE teaching mode according to the feedback information of decision tree. It can be seen from the data in the figure that after PE teachers adjusted the teaching contents and teaching methods according to the information fed back by the decision tree algorithm, the good rate of students has been greatly improved and the failure rate has decreased. Although the increase of excellence rate is small, the improvement of good rate lays a foundation for the improvement of excellence rate. This shows that the physical education teaching mode system based on the decision tree algorithm can effectively mine students' performance, behavior, and physical education teaching content and methods, find important influencing factors and the relationship between factors, and provide data support for teachers' adjustment of physical education teaching mode and targeted teaching.

The above discussion is only a beneficial attempt of the application of decision tree data mining technology in the field of physical education teaching in colleges and universities. Data mining refers to the automatic exploratory analysis of a large number of complex datasets by computer. The process of extracting implicit previously unknown and potentially valuable information, rules, and knowledge from massive, high-dimensional, uneven data quality, and random data. It is based on the theory and technology of artificial intelligence, machine learning, pattern recognition, mathematical statistics, database management, parallel computing, and other disciplines. The application of data is upgraded from low-level description and inference to mining knowledge from data, building prediction models and providing decision support. The essential characteristic of data mining technology, which is different from the traditional statistical data analysis, is to obtain the previously unknown, effective, and practical information, rules, and knowledge through data mining methods without explicit assumptions. The introduction of data mining technology into the research field of college physical education teaching will give fresh vitality to the development of college physical education.

## 5. Conclusion

This study puts forward the construction and analysis of discrete system dynamic modeling of physical education teaching mode based on the decision tree algorithm and analyzes and mines the relevant physical education teaching data through the constructed physical education teaching decision tree system. The test results show that the physical education teaching mode system based on the decision tree algorithm can analyze the given conditions and construct the corresponding decision tree according to the analysis results. The decision tree constructed in this study takes the number of students participating in sports competition as the root node, which shows that sports competition, as a comprehensive physical education teaching model, can play a targeted guiding role for students in a short time and help students correct their mistakes and make up for their deficiencies. Students' love of physical education and physical education teachers' physical education skills are secondary influencing factors. In addition, the diversity of physical education teachers' teaching means the number of physical education classes and students' own quality is closely related to students' physical education achievements. At the same time, according to the analysis results of physical education teaching decision tree, after the physical education teachers make the corresponding physical education teaching adjustment, the students' performance and before the adjustment have been improved to a certain extent, in which the excellent rate has been significantly improved and the unqualified rate has been significantly reduced. There are still some differences between the conditions of the decision tree test and the actual situation. The scale of basic data is relatively small. Therefore, further application testing is needed to improve the accuracy and reliability of decision tree.

The article "Construction and Analysis of Discrete System Dynamic Modeling of Physical Education Teaching Mode Based on Decision Tree Algorithm" was published in 2022. Journal: Comput Intell Neurosci.

## Figures and Tables

**Figure 1:** System framework of physical education teaching mode based on the decision tree algorithm.

**Figure 2:** Application structure of decision base of physical education teaching mode based on the decision tree algorithm.

**Figure 3:** Frame diagram of physical education decision tree based on knowledge point *K*_2_.

**Figure 4:** The tested eight attribute status statistics of some groups of the selected analysis variable training set.

**Figure 5:** Information gain and information gain rate of physical education decision tree.

**Figure 6:** Information gain and information gain rate of decision tree.

**Figure 7:** Comparison of students' achievements after the adjustment of physical education teaching mode.

## Data Availability

The data used to support the findings of this study are available from the corresponding author upon request.
